# Dynamics of a Fractional-Order Chikungunya Model with Asymptomatic Infectious Class

**DOI:** 10.1155/2022/5118382

**Published:** 2022-02-07

**Authors:** Mlyashimbi Helikumi, Gideon Eustace, Steady Mushayabasa

**Affiliations:** ^1^Mbeya University of Science and Technology, Department of Mathematics and Statistics, College of Science and Technical Education, P.O. Box 131, Mbeya, Tanzania; ^2^Department of Mathematics & Computational Sciences, University of Zimbabwe, P.O. Box MP 167, Harare, Zimbabwe

## Abstract

In this paper, a nonlinear fractional-order chikungunya disease model that incorporates asymptomatic infectious individuals is proposed and analyzed. The main interest of this work is to investigate the role of memory effects on the dynamics of chikungunya. Qualitative analysis of the model's equilibria showed that there exists a threshold quantity which governs persistence and extinction of the disease. Model parameters were estimated based on the 2015 weekly reported cases in Colombia. The Adams-Bashforth-Moulton method was used to numerically solve the proposed model. We investigated the role of asymptomatic infectious patients on short- and long-term dynamics of the diseases. We also determined threshold levels for the efficacy of preventative strategies that results in effective management of the disease. We believe that our model can provide invaluable insights for public health authorities to predict the effect of chikungunya transmission and analyze its underlying factors and to guide new control efforts.

## 1. Introduction

Emerging and reemerging diseases of vector-borne infections such as Zika virus and chikungunya pose a considerable public health problem worldwide [1]. Previous studies reported that vector-borne diseases are emerging at a growing rate and bearing a disproportionate segment of all new infectious diseases, the vast majority of them being viruses [1, 2]. These diseases are currently associated with high mortality and morbidity, which triggers immeasurable loss in many societies. For this reason, there is growing interest among researchers to utilize different techniques to study the dynamics of vector-borne infections with a goal to provide useful means for policymakers to evaluate potential ways of effectively managing these diseases [3, 4].

Although various techniques can be used to understand the short- and long-term dynamics of vector-borne infections, mathematical modeling is now regarded as a standard and indispensable tool for understanding the mechanisms of interaction between host and vectors [5, 6]. Models are used to approach questions which are too complex, inaccessible, numerous, diverse, mutable, unique, dangerous, expensive, big, small, slow, or fast to approach by other means [7]. In this study, we seek to develop and analyze a mathematical framework for understanding the dynamics of chikungunya virus.

Chikungunya is a viral infection whose causative agent is an alphavirus that infects humans through bites of Aedes mosquitoes [8]. The initial chikungunya cases were in Tanzania in the mid-1900s [9]. The clinical indications of chikungunya infections resemble those of dengue fever and include rashes and high fever [9, 10]. The onset of the disease in humans is often rapid and takes 5-7 days, and several case fatalities have been reported [11, 12]. Over the past 50 years, numerous cases of chikungunya reemergence have occurred in different parts of Africa and Asia [13, 14]. The infection has presently been established in nearly 40 countries but is endemic in Africa where its transmission is maintained between mosquitoes, primates, and humans [15]. The most notable outbreak occurred in India in 2005-2006 when the WHO approximated 1.3 million cases [16, 17].

In the last two decades, a plethora of mathematical models have been proposed to explain and predict as well as quantify the effectiveness ways of managing chikungunya virus (see, for example, [8, 18–26] and references therein). Yakob and Clements [8] constructed and analyzed a deterministic mathematical model for chikungunya virus that incorporated two infected human subpopulations designated as symptomatic and asymptomatic. Among several outcomes, their study demonstrated the strong influence that both the latent period of infection in humans and the prepatent period have on the dynamics of the disease. In [20], a spatial stochastic model was utilized to show that perifocal vector control is capable of limiting the spread of chikungunya. In [23], a stochastic model that incorporated climate-based mosquito population was proposed to identify temporal windows that have epidemic risk in the United States (US). Among several outcomes, their work strongly suggested that, in the event of an introduction and establishment of chikungunya in the US, endemic and epidemic regions would emerge initially, primarily defined by environmental factors controlling annual mosquito population cycles. In [24], a system of ordinary differential equations was employed to investigate and understand the importance of different model parameters on the dynamics of chikungunya. In [26], a mathematical framework was proposed to model and analyze virus mutation dynamics of chikungunya outbreaks. Results from their study suggested that the virus mutation dynamics could play an important role in the transmission of chikungunya. Hence, there is a need to better understand the mutation mechanism.

Despite these efforts, however, not much has been done to investigate the role of memory effects on chikungunya virus dynamics. Previous studies suggest that memory effects are inherent in many biological phenomena and models based on integer-order differentiation do not adequately capture the memory effects [27, 28]. Based on this assertion, fractional-order calculus has been widely and extensively used by several researchers recently, to investigate the role of memory effects in different diseases [29–33]. The fractional derivative has several definitions such as those derived from Riemann-Liouville, Caputo, Liouville, Weyl, Riesz, Grünwald-Litnikov, Marchaud and Hifler, Caputo-Fabrizio-Caputo, Atanga-Baleanu, Atanga-beta derivative, *𝕄*-fractional derivative, conformable derivative, Atangana-Koca, Atanga-Gomez, and variable-order and fractal-fractional idea [34, 35].

Motivated by the above-mentioned works, we derive a fractional-order model for chikungunya virus based on the Caputo derivative. The choice of using the Caputo derivative is also aided by the fact that the Caputo derivative for a given function which is constant is zero. Thus, the Caputo operator computes an ordinary differential equation, followed by a fractional integral to obtain the desired order of fractional derivative [36]. Most importantly, the Caputo fractional derivative allows the use of local initial conditions to be included in the derivation of the model [33, 36].

The remaining part of this paper is organized as follows: Section 2 contains some few basic definitions on fractional calculus. These definitions will be utilized to establish several important results. In Section 3, we propose and qualitatively analyze a fractional-order chikungunya virus model. In particular, we computed the reproduction number and demonstrated that it is an important threshold quantity for disease persistence and extinction.  Section 4 contains numerical illustrations and discussions. The paper is concluded in Section 5

## 2. Preliminaries on Fractional Calculus

Throughout the paper, we use the Caputo fractional-order derivatives because the initial conditions of fractional differential equations with Caputo derivative take on the same form as that of the integer-order ones, which have received more attention in modeling and analysis of many real-world phenomena despite their inability to capture memory effects, which are inherent in these phenomena. In this section, we will present some essential definitions and lemmas that will be utilized to determine the dynamical behavior of the proposed model.

**Definition 1 (see [37]).**

*The Riemann-Liouville fractional integral operator of orderθof a continuous functionf* : [*t*_0_, +∞)⟶ℝ*is defined as*

(1) $$\begin{array}{c} I^{\theta }f\left(t\right)=\frac{1}{\Gamma \left(\theta \right)}\int_{0}^{t}{\left(t-s\right)}^{\theta -1}f\left(s\right)ds, \end{array}$$

where Γ(·) is the gamma function and is defined by Γ(*z*) = ∫_0_^∞^*e*^−*t*^*t*^*z*−1^*dt* and *θ* > 0.

**Definition 2 (see [37]).**

*The Caputo fractional derivative of orderθfor a functionf* ∈ *C*^*n*^([*t*_0_, +∞), ℝ)*is defined by*

(2) $$\begin{array}{c} {\;}_{t_{0}}^{c}D_{t}^{\theta }f\left(t\right)=\frac{1}{\Gamma \left(n-\theta \right)}\int_{t_{0}}^{t}\frac{f^{\left(n\right)}\left(s\right)}{{\left(t-s\right)}^{\theta -n+1}}ds, \end{array}$$

where *t* ≥ *t*_0_ and *n* is a positive integer such that *n* − 1 < *θ* < *n* ∈ *ℕ*. In particular, if 0 < *θ* < 1, then the Caputo fractional derivative takes the form

(3) $$\begin{array}{c} {\;}_{b}^{c}D_{t}^{\theta }f\left(t\right)=\frac{1}{\Gamma \left(1-\theta \right)}\int_{t_{0}}^{t}\frac{f^{\prime }\left(s\right)}{{\left(t-s\right)}^{\theta }}ds. \end{array}$$

**Lemma 1 (see [38]).**

*The solution to the Cauchy problem*

(4) Dtθt0cxt=λxt+ft,xa=bb∈ℝ

with 0 < *θ* < 1 and *λ* ∈ ℝ has the form

(5) $$\begin{array}{c} x\left(t\right)=bE_{\theta }\left[\lambda {\left(t-a\right)}^{\theta }\right]+\int_{a}^{t}{\left(t-s\right)}^{\theta -1}E_{\theta ,\theta }\left[\lambda {\left(t-s\right)}^{\theta }\right]f\left(s\right)ds, \end{array}$$

while the solution to the problem

(6) Dtθt0cxt=λxt,xa=bb∈ℝ

is given by

(7) $$\begin{array}{c} x\left(t\right)=bE_{\theta }\left[\lambda {\left(t-a\right)}^{\theta }\right], \end{array}$$

where *E*_*θ*_(·) is the Mittag-Leffler function and defined by

(8) $$\begin{array}{c} E_{\theta }\left(z\right)=\overset{\infty }{\underset{k=0}{\sum }}\frac{z^{k}}{\Gamma \left(\theta k+1\right)},\;\theta >0,z\in \mathbb{C}. \end{array}$$

**Lemma 2 (see [39]).**

*Letu*(*t*)*be a continuous function on*[*t*_0_, +∞)*and satisfying*

(9) Dtθt0cut=−λut+μ,ut0=ut0,

with 0 < *θ* < 1, (*λ*, *μ*) ∈ ℝ^2^, and *λ* ≠ 0, and *t*_0_ ≥ 0 is the initial time. Then,

(10) $$\begin{array}{c} u\left(t\right)\leq \left(u_{t_{0}}-\frac{\mu }{\lambda }\right)E_{\theta }\left[-\lambda {\left(t-t_{0}\right)}^{\theta }\right]+\frac{\mu }{\lambda }. \end{array}$$

**Lemma 3 (see [40]).**

*Letx*(*t*)*be a continuous and differentiable function withx*(*t*) ∈ ℝ_+_*. Then, for any time instantt* ≥ *t*_0_*, one has*

(11) $$\begin{array}{c} {\;}_{t_{0}}^{c}D_{t}^{\theta }\left[x\left(t\right)-x^{*}-x^{*}\ln\frac{x\left(t\right)}{x^{*}}\right]\leq {\left(1-\frac{x^{*}}{x\left(t\right)}\right)}_{t_{0}}^{c}D_{t}^{\theta }x\left(t\right),\;x^{*}\in {\mathbb{R}}^{+},\forall \theta \in \left(0,1\right). \end{array}$$

## 3. Model Formulation and Analytical Results

### 3.1. Model Formulation

Owing to the merits of fractional derivatives (discussed in Introduction) in modeling real-world problems in comparison to integer ordinary differential equations, in this section, we propose a fractional-order model for chikungunya infection. The proposed model (12) is based on the Caputo fractional operator which is known to be the most suitable for modeling biological and physical phenomena [36]. The proposed model is governed by the following assumptions:

- The total populations of humans *N*_*h*_(*t*) are subdivided into classes of susceptible *S*_*h*_(*t*), exposed *E*_*h*_(*t*), asymptomatic infectious individuals *A*_*h*_(*t*), symptomatic infectious individuals *I*_*h*_(*t*), and humans who have recovered from infection *R*_*h*_(*t*). The total vector population *N*_v_(*t*) is subdivided into compartments of susceptible *S*_*v*_(*t*), exposed *E*_*v*_(*t*), and infectious *I*_*v*_(*t*). Once infected, vectors are assumed to remain infectious for their entire life span. Throughout this paper, we will use the subscripts *h* and *v* to represent the human and vector population, respectively
- Disease transmission is assumed to occur solely when there is interaction between the host and vector. Thus, all new recruits in the both the host and vector are assumed to be susceptible to infection. In most cases, chikungunya disease does not lead to death, but its symptoms can be severe and disabling [41]. Based on this assertion, we assumed a constant size population in both the host and vector with a recruitment and non-disease-related mortality rate modeled by *μ*_*j*_ with *j* = *h*, *v*. Further, new recruits are assumed susceptible and their recruitment rate is proportional to the population and is given by *μ*_*j*_*N*_*j*_. Meanwhile, we assume that whenever there is effective contact between a susceptible individual and an infectious vector, disease transmission will occur at rate *β*_*v*_. Similarly, let *β*_*h*_ be the transmission rate of the disease from a infectious human to a susceptible vector whenever there is effective contact. Asymptomatic infectious individuals are assumed to have less parasite load compared to symptomatic infectious individuals. To account for this aspect, in our model formulation, we introduce a factor (1 − *η*_*h*_) to model the reduction of infectivity of the asymptomatic individuals
- Although there is no vaccine to prevent chikungunya virus infection, humans can minimize chances of contracting the infections through a number of strategies such as the use of insect repellent, wearing of long-sleeved shirts and pants, and treating clothing and gear. Let 1 − *ε*_*h*_ model the effects of preventative strategies utilized by humans to minimize chances of contracting the infection (naturally or through treatment)
- Exposed humans are assumed to incubate the infection for 1/*α*_*h*_ days after which a proportion *f*_*h*_ become asymptomatic infectious patients and the remainder, (1 − *f*_*h*_), become symptomatic infectious patients. The average infectious period of asymptomatic infectious individuals is modeled by 1/*γ*_*h*_, and symptomatic infectious individuals are assumed to be infectious for an average period of 1/*σ*_*h*_ days
- Exposed vectors incubate the disease for 1/*α*_*v*_ days after which they become infectious. Once infected, vectors are assumed to remain infectious for their entire life span

Based on the above assumptions, the proposed model (12) is summarized in Figure 1 and akes the following form:

(12) $$\begin{array}{c} \left.\begin{array}{c} {\;}_{b}^{c}D_{t}^{\theta }S_{h}\left(t\right)=\mu_{h}N_{h}\left(t\right)-\frac{\left(1-\varepsilon_{h}\right)\beta_{v}cI_{v}\left(t\right)}{N_{h}\left(t\right)}S_{h}\left(t\right)-\mu_{h}S_{h}\left(t\right),\\ {\;}_{b}^{c}D_{t}^{\theta }E_{h}\left(t\right)=\frac{\left(1-\varepsilon_{h}\right)\beta_{v}cI_{v}\left(t\right)}{N_{h}\left(t\right)}S_{h}\left(t\right)-\left(\alpha_{h}+\mu_{h}\right)E_{h}\left(t\right),\\ \begin{array}{c} {\;}_{b}^{c}D_{t}^{\theta }A_{h}\left(t\right)=f_{h}\alpha_{h}E_{h}\left(t\right)-\left(\mu_{h}+\gamma_{h}\right)A_{h}\left(t\right),\\ {\;}_{b}^{c}D_{t}^{\theta }I_{h}\left(t\right)=\left(1-f_{h}\right)\alpha_{h}E_{h}\left(t\right)-\left(\mu_{h}+\sigma_{h}\right)I_{h}\left(t\right),\\ \begin{array}{c} {\;}_{b}^{c}D^{\theta }R_{h}\left(t\right)=\gamma_{h}A_{h}\left(t\right)+\sigma_{h}I_{h}\left(t\right)-\mu_{h}R_{h}\left(t\right),\\ {\;}_{b}^{c}D_{t}^{\theta }S_{v}\left(t\right)=\mu_{v}N_{v}\left(t\right)-\frac{\left(1-\varepsilon_{h}\right)\beta_{h}c\left[I_{h}\left(t\right)+\left(1-\eta_{h}\right)A_{h}\left(t\right)\right]}{N_{h}\left(t\right)}S_{v}\left(t\right)-\mu_{v}S_{v}\left(t\right),\\ \begin{array}{c} {\;}_{b}^{c}D_{t}^{\theta }E_{v}\left(t\right)=\frac{\left(1-\varepsilon_{h}\right)\beta_{h}c\left[I_{h}\left(t\right)+\left(1-\eta_{h}\right)A_{h}\left(t\right)\right]}{N_{h}\left(t\right)}S_{v}\left(t\right)-\left(\alpha_{v}+\mu_{v}\right)E_{v}\left(t\right),\\ {\;}_{b}^{c}D_{t}^{\theta }I_{v}\left(t\right)=\alpha_{v}E_{v}\left(t\right)-\mu_{v}I_{v}\left(t\right), \end{array} \end{array} \end{array} \end{array}\right\} \end{array}$$

where *θ* ∈ (0, 1] is the order of the fractional derivative. Model (12) is subject to the initial conditions:

(13) $$\begin{array}{c} S_{j}\left(0\right)=S_{j0},\\ E_{j}\left(0\right)=E_{j0},\\ A_{h}\left(0\right)=A_{h0},\\ I_{j}\left(0\right)=I_{j0},\\ R_{h}\left(0\right)=R_{h0}, \end{array}$$

for *j* = *h*, *v*. By adding all the equations that govern the dynamics of the disease in the host, one can observed that the human population is assumed to be constant. Similarly, by adding all the equations for the vector population, one can also observe that the vector population is assumed to be constant. Based on this, we can consider normalized populations for both the vector and host. Let

(14) $$\begin{array}{c} s_{j}\left(t\right)=\frac{S_{j}\left(t\right)}{N_{j}\left(t\right)},\\ e_{j}\left(t\right)=\frac{E_{j}\left(t\right)}{N_{j}\left(t\right)},\\ i_{j}\left(t\right)=\frac{I_{j}\left(t\right)}{N_{j}\left(t\right)},\\ a_{h}\left(t\right)=\frac{A_{h}\left.t\right)}{N_{h}\left(t\right)},\\ r_{h}\left(t\right)=\frac{R_{h}\left(t\right)}{N_{h}\left(t\right)},\\ \phi =\frac{N_{v}\left(t\right)}{N_{h}\left(t\right)}. \end{array}$$

Using the definitions in (18), the chikungunya model with normalized populations is given as follows:

(15) $$\begin{array}{c} \left.\begin{array}{c} {\;}_{b}^{c}D_{t}^{\theta }s_{h}\left(t\right)=\mu_{h}-\left(1-\varepsilon_{h}\right)\beta_{v}\phi ci_{v}s_{h}-\mu_{h}s_{h},\\ {\;}_{b}^{c}D_{t}^{\theta }e_{h}\left(t\right)=\left(1-\varepsilon_{h}\right)\beta_{v}\phi ci_{v}s_{h}-m_{1}e_{h},\\ \begin{array}{c} {\;}_{b}^{c}D_{t}^{\theta }a_{h}\left(t\right)=f_{h}\alpha_{h}e_{h}-m_{2}a_{h},\\ {\;}_{b}^{c}D_{t}^{\theta }i_{h}\left(t\right)=\left(1-f_{h}\right)\alpha_{h}e_{h}-m_{3}i_{h},\\ \begin{array}{c} {\;}_{b}^{c}D^{\theta }r_{h}\left(t\right)=\gamma_{h}a_{h}+\sigma_{h}i_{h}-\mu_{h}r_{h},\\ {\;}_{b}^{c}D_{t}^{\theta }s_{v}\left(t\right)=\mu_{v}-\left(1-\varepsilon_{h}\right)\beta_{h}c\left[i_{h}+\left(1-\eta_{h}\right)a_{h}\right]s_{v}-\mu_{v}s_{v},\\ \begin{array}{c} {\;}_{b}^{c}D_{t}^{\theta }e_{v}\left(t\right)=\left(1-\varepsilon \right)\beta_{h}c\left[i_{h}+\left(1-\eta_{h}\right)a_{h}\right]s_{v}-m_{4}e_{v},\\ {\;}_{b}^{c}D_{t}^{\theta }i_{v}\left(t\right)=\alpha_{v}e_{v}-\mu_{v}i_{v}, \end{array} \end{array} \end{array} \end{array}\right\} \end{array}$$

with

(16) $$\begin{array}{c} m_{1}=\left(\alpha_{h}+\mu_{h}\right),\\ m_{2}=\left(\mu_{h}+\gamma_{h}\right),\\ m_{3}=\left(\mu_{h}+\sigma_{h}\right),\\ m_{4}=\left(\alpha_{v}+\mu_{v}\right), \end{array}$$

subject to the initial conditions

(17) $$\begin{array}{c} s_{j}\left(0\right)=s_{j0},\\ e_{j}\left(0\right)=e_{j0},\\ a_{h}\left(0\right)=a_{j0},\\ i_{j}\left(0\right)=i_{j0},\\ r_{h}\left(0\right)=r_{h0}, \end{array}$$

for *j* = *h*, *v*. Since the variable *r*_*h*_(*t*) does not appear in any other equations of system (12), it suffices to analyze the dynamics of chikungunya virus infection from the following reduced system:

(18) $$\begin{array}{c} \left.\begin{array}{c} {\;}_{b}^{c}D_{t}^{\theta }s_{h}\left(t\right)=\mu_{h}-\left(1-\varepsilon_{h}\right)\beta_{v}\phi ci_{v}s_{h}-\mu_{h}s_{h},\\ {\;}_{b}^{c}D_{t}^{\theta }e_{h}\left(t\right)=\left(1-\varepsilon_{h}\right)\beta_{v}\phi ci_{v}s_{h}-m_{1}e_{h},\\ \begin{array}{c} {\;}_{b}^{c}D_{t}^{\theta }a_{h}\left(t\right)=f_{h}\alpha_{h}e_{h}-m_{2}a_{h},\\ {\;}_{b}^{c}D_{t}^{\theta }i_{h}\left(t\right)=\left(1-f_{h}\right)\alpha_{h}e_{h}-m_{3}i_{h},\\ \begin{array}{c} {\;}_{b}^{c}D_{t}^{\theta }s_{v}\left(t\right)=\mu_{v}-\left(1-\varepsilon \right)\beta_{h}c\left(i_{h}+\left(1-\eta_{h}\right)a_{h}\right)s_{v}-\mu_{v}s_{v},\\ {\;}_{b}^{c}D_{t}^{\theta }e_{v}=\left(1-\varepsilon \right)\beta_{h}c\left(i_{h}+\left(1-\eta_{h}\right)a_{h}\right)s_{v}-m_{4}e_{v},\\ {\;}_{b}^{c}D_{t}^{\theta }i_{v}\left(t\right)=\alpha_{v}e_{v}-\mu_{v}i_{v}. \end{array} \end{array} \end{array}\right\} \end{array}$$

### 3.2. Positivity and Boundedness of Model Solutions

**Theorem 1 .**

*The fractional order* (18) *has a unique solution, which remains in*ℝ^7^, *and the closed set*

(19) $$\begin{array}{c} \Omega =\left\{\left(\begin{array}{c} s_{h},e_{h},a_{h},i_{h}\\ s_{v},e_{v},i_{v} \end{array}\right)\in {\mathbb{R}}_{+}^{7}\left|\begin{array}{c} s_{h}\geq 0,e_{h}\geq 0,a_{h}\geq 0,i_{h}\geq 0\\ s_{h}+e_{h}+a_{h}+i_{h}\leq 1\\ s_{v}\geq 0,e_{v}\geq 0,i_{v}\geq 0\\ s_{v}+e_{v}+i_{v}\leq 1 \end{array}\right.\right\} \end{array}$$

is a positive invariant set of system (18).

**Proof**

We begin by demonstrating that the solution of system (18) is always nonnegative for all *t* ≥ 0. Based on system (18), we have (for *j* = *h*, *v*)

(20) $$\begin{array}{c} \left.\begin{array}{c} {\left.{\;}_{t_{0}}^{c}D_{t}^{\theta }s_{h}\left(t\right)\right|}_{s_{j}=0}=\mu_{j}\geq 0,\\ {\left.{\;}_{t_{0}}^{c}D_{t}^{\theta }e_{h}\left(t\right)\right|}_{e_{h}=0}=\left(1-\varepsilon_{h}\right)\beta_{v}\phi ci_{v}s_{h}\geq 0,\\ \begin{array}{c} {\left.{\;}_{t_{0}}^{c}D_{t}^{\theta }a_{h}\left(t\right)\right|}_{a_{h}=0}=f_{h}\alpha_{h}e_{h}\geq 0,\\ {\left.{\;}_{t_{0}}^{c}D_{t}^{\theta }i_{h}\left(t\right)\right|}_{i_{h}=0}=\left(1-f_{h}\right)\alpha_{h}e_{h}\geq 0,\\ \begin{array}{c} {\left.{\;}_{t_{0}}^{c}D_{t}^{\theta }\left(t\right)\right|}_{e_{v}=0}=\left(1-\varepsilon_{h}\right)\beta_{h}c\left(i_{h}+\left(1-\eta_{h}\right)a_{h}\right)s_{v}\geq 0,\\ {\left.{\;}_{t_{0}}^{c}D_{t}^{\theta }i_{v}\left(t\right)\right|}_{i_{v}=0}=\alpha_{v}e_{v}\geq 0. \end{array} \end{array} \end{array}\right\} \end{array}$$

Results in equation (20) demonstrate that the vector field given by the right-hand side of (18) on each coordinate plane either is tangent to the coordinate plane or points to the interior of ℝ_+_^7^. Hence, the domain ℝ_+_^7^ is a positively invariant region. Moreover, if the initial conditions of system (18) are nonnegative, then it follows that the corresponding solutions of model (18) are nonnegative. Let *n*_*h*_(*t*) = *s*_*h*_(*t*) + *e*_*h*_(*t*) + *a*_*h*_(*t*) + *i*_*h*_(*t*). By adding all the equations for the host population in (6), one gets

(21) $$\begin{array}{c} {\;}_{t_{0}}^{c}D_{t}^{\theta }n_{h}\left(t\right)\leq \mu_{h}-\mu_{h}n_{h}. \end{array}$$

It follows from Lemma 3 that (38) has a solution of the form

(22) $$\begin{array}{c} n_{h}\left(t\right)\leq \left(n_{h}\left(0\right)-1\right)E_{\theta }\left(-\mu_{h}t^{\theta }\right)+1. \end{array}$$

Since *E*_*θ*_(−*μ*_*h*_*t*^*θ*^) ≥ 0, so that when *n*_*h*_(0) ≤ 1, we have *n*_*h*_(*t*) ≤ 1. Similarly, by adding all the equations for the vector population (with, *n*_*v*_ = *s*_*v*_ + *e*_*v*_ + *i*_*v*_), one gets

(23) $$\begin{array}{c} {\;}_{t_{0}}^{c}D_{t}^{\theta }n_{v}\left(t\right)=\mu_{v}-\mu_{v}n_{v}. \end{array}$$

Again, by Lemma 3, we have

(24) $$\begin{array}{c} n_{v}\left(t\right)\leq \left(n_{v}\left(0\right)-1\right)E_{\theta }\left(-\mu_{v}t^{\theta }\right)+1. \end{array}$$

By similar arguments as before, we have *n*_*v*_(*t*) ≤ 1. This completes the proof.☐

### 3.3. Model Equilibria, Their Existence, and Global Stability

Direct calculations of system (18) show that the proposed model admits two equilibrium points, namely, the disease-free equilibrium (DFE) point (denoted by *E*^0^) and the endemic equilibrium (EE) point (denoted by *E*^∗^) point, which are, respectively, given by *E*^0^ : (*s*_*h*_^0^, *e*_*h*_^0^, *a*_*h*_^0^, *i*_*h*_^0^, *s*_*v*_^0^, *e*_*v*_^0^, *i*_*v*_^0^) = (1, 0, 0, 0, 1, 0, 0). The endemic equilibrium (EE) point *E*^∗^ = (*S*_*h*_^∗^, *E*_*h*_^∗^, *I*_*h*_^∗^, *S*_*v*_^∗^, *E*_*v*_^∗^, *I*_*v*_^∗^) with

(25) $$\begin{array}{c} \left.\begin{array}{c} s_{h}^{*}=\frac{m_{4}\left(\beta_{h}\right.\left(1-\varepsilon_{h}\right)c\alpha_{h}\mu_{h}\left(\left(1-f_{h}\right)m_{2}+\left(1-\eta_{h}\right)f_{h}m_{3}\right)}{H_{1}},\\ e_{h}^{*}=\frac{\mu_{v}\mu_{h}m_{2}m_{3}m_{4}}{H_{1}}\left(R_{0}^{2}-1\right),a_{h}^{*}=\frac{\mu_{v}\mu_{h}m_{3}m_{4}f_{h}\alpha_{h}}{H_{1}}\left(R_{0}^{2}-1\right),\\ \begin{array}{c} i_{h}^{*}=\frac{\mu_{v}\mu_{h}m_{2}m_{4}\left(1-f_{h}\right)\alpha_{h}}{H_{1}}\left(R_{0}^{2}-1\right),s_{v}^{*}=\frac{\mu_{v}m_{1}m_{2}m_{3}\left(\beta_{v}\left(1-\varepsilon_{h}\right)\phi c\alpha_{v}+\mu_{h}m_{4}\right)}{H_{2}},\\ e_{v}^{*}=\frac{\mu_{v}^{2}\mu_{h}m_{1}m_{2}m_{3}}{\beta_{v}\left(1-\varepsilon \right)\phi c\alpha_{v}H_{2}}\left(R_{0}^{2}-1\right)i_{v}^{*}=\frac{\mu_{v}\mu_{h}m_{1}m_{2}m_{3}}{\beta_{v}\left(1-\varepsilon_{h}\right)\phi cH_{2}}\left(R_{0}^{2}-1\right), \end{array} \end{array}\right\} \end{array}$$

with

(26) $$\begin{array}{c} H_{1}=\beta_{h}c\left(1-\varepsilon_{h}\right)\alpha_{h}\left(\beta_{v}\phi \left(1-\varepsilon_{h}\right)c\alpha_{v}+\mu_{h}m_{4}\right)\left(\left(1-f_{h}\right)m_{2}+\left(1-\eta \right)f_{h}m_{3}\right),\\ H_{2}=\left(1-f_{h}\right)m_{2}\alpha_{h}\beta_{h}\left(1-\varepsilon_{h}\right)c\mu_{h}+m_{3}\left[\left(1-\eta \right)f_{h}\alpha_{h}\left(1-\varepsilon_{h}\right)\beta_{h}\mu_{h}+m_{1}m_{2}\mu_{v}\right],\\ R_{0}=\sqrt{\frac{\beta_{v}\beta_{h}\phi c^{2}{\left(1-\varepsilon_{h}\right)}^{2}\alpha_{v}\alpha_{h}}{\mu_{v}m_{1}m_{4}}\left(\frac{\left(1-\eta_{h}\right)f_{h}}{m_{2}}+\frac{\left(1-f_{h}\right)}{m_{3}}\right)}. \end{array}$$

In equation (25), we can note that the disease persists in the community if *R*_0_ > 1. Precisely, the threshold quantity *R*_0_ demonstrates the power of the disease to persist or become extinct in the host population. Thus, the expression *R*_0_ defines the basic reproduction number of the proposed fractional-order model.

**Theorem 2 .**

*IfR*_0_ < 1*, then the DFE of system (*(18)*) is globally asymptotically stable inΩ, otherwise it is unstable.*

**Proof**

By considering only the infected compartments from (18), we can write

(27) $$\begin{array}{c} {\;}_{b}^{c}D_{t}^{\theta }x=\left(F-V\right)x, \end{array}$$

where *x* = (*e*_*h*_, *a*_*h*_, *i*_*h*_, *e*_*v*_, *i*_*v*_)^*T*^, with *F* and *V* defined as follows:

(28) $$\begin{array}{c} F=\left[\begin{array}{ccccc} 0 & 0 & 0 & 0 & \beta_{v}\left(1-\varepsilon \right)\theta c\\ 0 & 0 & 0 & 0 & 0\\ 0 & 0 & 0 & 0 & 0\\ 0 & \beta_{h}\left(1-\varepsilon \right)\left(1-\eta \right)c & \beta_{h}\left(1-\varepsilon \right)c & 0 & 0\\ 0 & 0 & 0 & 0 & 0 \end{array}\right],\\ V=\left[\begin{array}{ccccc} m_{1} & 0 & 0 & 0 & 0\\ -f_{h}\alpha_{h} & m_{2} & 0 & 0 & 0\\ -\left(1-f_{h}\right)\alpha_{h} & 0 & m_{3} & 0 & 0\\ 0 & 0 & 0 & m_{4} & 0\\ 0 & 0 & 0 & -\alpha_{v} & \mu_{v} \end{array}\right]. \end{array}$$

One can verify by direct calculations that *V*^−1^*F* is a nonnegative and irreducible matrix and *ρ*(*V*^−1^*F*) = *R*_0_. It follows from the Perron-Frobenius theorem [42] that *V*^−1^*F* has positive left eigenvector **w** associated with *R*_0_, i.e.,

(29) $$\begin{array}{c} wV^{-1}F=R_{0}w. \end{array}$$

Since **w***V*^−1^ is a positive vector, we propose the following Lyapunov function to study the global stability of DFE:

(30) $$\begin{array}{c} L\left(t\right)=wV^{-1}x. \end{array}$$

Differentiating *L* along solutions of (12) leads to

(31) $$\begin{array}{c} {\;}_{b}^{c}D_{t}^{\theta }L\left(t\right)=w{V^{-1}}_{b}^{c}D_{t}^{\theta }x\leq wV^{-1}\left(F-V\right)x=\left(R_{0}-1\right)wx\leq 0\;\text{if }R_{0}\leq 1. \end{array}$$

It can be easily verified that the largest invariant subset of Γ where  _*b*_^*c*^*D*_*t*_^*θ*^*L*(*t*) = 0 is the singleton {*ℰ*^0^}. Therefore, by LaSalle's invariance principle [43], *ℰ*^0^ is globally asymptotically stable in Γ when *R*_0_ ≤ 1.☐

**Theorem 3 .**

*IfR*_0_ > 1, *then the endemic equilibriumE*^∗^*of system (*(18)*) is globally asymptotically stable inΩ*.

**Proof**

To prove Theorem 8, we consider the following Lyapunov functional:

(32) $$\begin{array}{c} U\left(t\right)=\left(s_{h}-s_{h}^{*}-s_{h}^{*}\ln\frac{s_{h}}{s_{h}^{*}}\right)+\left(e_{h}-e_{h}^{*}-e_{h}^{*}\ln\frac{e_{h}}{e_{h}^{*}}\right)+w_{1}\left(a_{h}-a_{h}^{*}-a_{h}^{*}\ln\frac{a_{h}}{a_{h}^{*}}\right)w_{2}\left(i_{h}-i_{h}^{*}-i_{h}^{*}\ln\frac{i_{h}}{i_{h}^{*}}\right)+w_{3}\left(s_{v}-s_{v}^{*}-s_{v}^{*}\ln\frac{s_{v}}{s_{v}^{*}}\right)+w_{3}\left(e_{v}-e_{v}^{*}-e_{v}^{*}\ln\frac{e_{v}}{e_{v}^{*}}\right)+w_{4}\left(i_{v}-i_{v}^{*}-i_{v}^{*}\ln\frac{i_{v}}{i_{v}^{*}}\right). \end{array}$$

Let *g*(*i*_*h*_, *a*_*h*_) = *i*_*h*_ + *η*_*h*_*a*_*h*_. At the endemic equilibrium, we have the following identities:

(33) $$\begin{array}{c} \mu_{h}=\left(1-\varepsilon \right)\beta_{v}\phi ci_{v}^{*}s_{h}^{*}+\mu_{h}s_{h}^{*}m_{1}e_{h}^{*}=\left(1-\varepsilon \right)\beta_{v}\phi ci_{v}^{*}s_{h}^{*},m_{2}a_{h}^{*}=f_{h}\alpha_{h}e_{h}^{*},m_{3}i_{h}^{*}=\left(1-f_{h}\right)\alpha_{h}e_{h}^{*},\mu_{v}=\left(1-\varepsilon \right)\beta_{h}cg\left(i_{h}^{*},a_{h}^{*}\right)s_{v}^{*}-\mu_{v}s_{v}^{*},m_{4}e_{v}^{*}=\left(1-\varepsilon \right)\beta_{h}g\left(i_{h}^{*},a_{h}^{*}\right)s_{v}^{*},\mu_{v}i_{v}^{*}=\alpha_{v}e_{v}^{*}. \end{array}$$

Let

(34) $$\begin{array}{c} w_{1}=\frac{\beta_{v}i_{v}^{*}s_{h}^{*}}{\left(1-f_{h}\right)\alpha_{h}e_{h}^{*}},\\ w_{2}=\frac{\beta_{v}i_{v}^{*}s_{h}^{*}}{f_{h}\alpha_{h}e_{h}^{*}},\\ w_{3}=\frac{\beta_{v}i_{v}^{*}s_{h}^{*}}{\beta_{h}g\left(i_{h}^{*},a_{h}^{*}\right)s_{v}^{*}},\\ w_{4}=\frac{\beta_{v}i_{v}^{*}s_{h}^{*}}{\alpha_{v}e_{v}^{*}}. \end{array}$$

After some algebraic manipulations, one gets

(35) $$\begin{array}{c} {\;}_{t_{0}}^{c}DU\left(t\right)\leq \mu_{h}\left(2-\frac{s_{h}}{s_{h}^{*}}-\frac{s_{h}^{*}}{s_{h}}\right)+\mu_{v}w_{3}\left(2-\frac{S_{v}}{S_{v}^{*}}-\frac{S_{v}^{*}}{S_{v}}\right)+\beta_{v}i_{v}^{*}s_{h}^{*}\left(7-\frac{s_{h}^{*}}{s_{h}}-\frac{s_{h}e_{h}^{*}i_{v}}{s_{h}^{*}e_{h}i_{v}^{*}}-\frac{a_{h}}{a_{h}^{*}}-\frac{e_{h}a_{h}^{*}}{e_{h}^{*}a_{h}}+\frac{e_{h}}{e_{h}^{*}}-\frac{e_{h}i_{h}^{*}}{e_{h}^{*}i_{h}}-\frac{i_{h}}{i_{h}^{*}}-\frac{s_{v}^{*}}{s_{v}}+\frac{g\left(i_{h},a_{h}\right)}{g\left(i_{h}^{*},a_{h}^{*}\right)}-\frac{s_{v}e_{v}g\left(i_{h}^{*},a_{h}^{*}\right)}{s_{v}^{*}e_{v}^{*}g\left(i_{h}^{*},a_{h}^{*}\right)}-\frac{e_{v}i_{v}^{*}}{e_{v}^{*}i_{v}}\right). \end{array}$$

Since the arithmetic mean is greater than or equal to the geometric mean, it follows that terms in the brackets are

(36) $$\begin{array}{c} 2\leq \frac{s_{j}}{s_{i}^{0}}+\frac{s_{i}^{0}}{s_{i}}\;j=h,v,7\leq \frac{s_{h}^{*}}{s_{h}}+\frac{s_{h}e_{h}^{*}i_{v}}{s_{h}^{*}e_{h}i_{v}^{*}}+\frac{a_{h}}{a_{h}^{*}}+\frac{e_{h}a_{h}^{*}}{e_{h}^{*}a_{h}}-\frac{e_{h}}{e_{h}^{*}}+\frac{e_{h}i_{h}^{*}}{e_{h}^{*}i_{h}}+\frac{i_{h}}{i_{h}^{*}}+\frac{s_{v}^{*}}{s_{v}}-\frac{g\left(i_{h},a_{h}\right)}{g\left(i_{h}^{*},a_{h}^{*}\right)}+\frac{s_{v}e_{v}g\left(i_{h}^{*},a_{h}^{*}\right)}{s_{v}^{*}e_{v}^{*}g\left(i_{h}^{*},a_{h}^{*}\right)}+\frac{e_{v}i_{v}^{*}}{e_{v}^{*}i_{v}}. \end{array}$$

Hence, we conclude that  _*t*_0__^*c*^*DU*(*t*) ≤ 0 for all (*s*_*h*_, *e*_*h*_, *a*_*h*_, *i*_*h*_, *s*_*v*_, *e*_*v*_, *i*_*v*_) ≥ 0 since *s*_*h*_^∗^, *e*_*h*_^∗^, *a*_*h*_^∗^, *i*_*h*_^∗^*s*_*v*_^∗^, *e*_*v*_^∗^, and *i*_*v*_^∗^ are nonnegative whenever *R*_0_ > 1. Therefore, by Lasalle's invariance principle [43], the endemic equilibrium point is globally asymptotically stable whenever *R*_0_ > 1.☐

## 4. Numerical Results and Discussions

In this section, we will make use of MATLAB programming language to simulate model (18) so as to support analytical findings and determine the implications of time-dependent controls. To simulate model (12), we make use of the technique so-called generalized Adams-Bashforth-Moulton (ABM) method [36]. For any nonlinear fractional differential equation,

(37) $$\begin{array}{c} {\;}_{b}^{c}D_{t}^{\theta }\psi \left(t\right)=f\left(t,\psi \left(t\right)\right),\;0\leq t\leq T, \end{array}$$

with the following initial conditions:

(38) $$\begin{array}{c} \psi^{m}\left(0\right)=\psi_{0}^{m},\;m=0,1,2,3,\cdots ,\left[\theta \right]-1. \end{array}$$

Now, with operating by the fractional integral operator on equation (37), we can obtain on the solution *ψ*(*t*) by solving the following equation:

(39) $$\begin{array}{c} \psi \left(t\right)=\overset{\left[\theta \right]-1}{\underset{m=0}{\sum }}\frac{\psi_{0}^{m}}{m!}t^{m}+\frac{1}{\Gamma \left(\theta \right)}\int_{0}^{t}{\left(t-\tau \right)}^{\theta -1}f\left(\tau ,\psi \left(\tau \right)\right)d\tau . \end{array}$$

Diethelm [44] used the predictor-corrector scheme based on the ABM algorithm to numerically solve (39). Setting *h* = *T*/*N*, *t*_*n*_ = *nh*, and *n* = 0, 1, 2, ⋯, *N* ∈ *ℤ*^+^, equation (39) can be discretized as follows:

(40) $$\begin{array}{c} \psi_{h}\left(t_{n+1}\right)=\overset{\;|\;\theta \;|\;-1}{\underset{m=0}{\sum }}\frac{\psi_{0}^{m}}{m!}t_{n+1}^{m}+\frac{h^{\theta }}{\Gamma \left(\theta +2\right)}\overset{n}{\underset{q=0}{\sum }}a_{q,n+1}f\left(t_{q},\psi_{q}\right)+\frac{h^{\theta }}{\Gamma \left(\theta +2\right)}f\left(t_{n+1},\psi_{n+1}^{p}\right), \end{array}$$

where

(41) $$\begin{array}{c} a_{q,n+1}=\left\{\begin{array}{cc} n^{\theta +1}-\left(n-\theta \right){\left(n+\theta \right)}^{\theta }, & q=0,\\ {\left(n-q+2\right)}^{\theta +1}+{\left(n-q\right)}^{\theta +1}-2{\left(n-q+1\right)}^{\theta +1}, & 1\leq q\leq n,\\ 1, & \text{if }q=n+1, \end{array}\right. \end{array}$$

and the predicted value *ψ*_*h*_^*p*^(*t*_*n*+1_) is determined by

(42) $$\begin{array}{c} \psi_{t_{n+1}}^{p}=\overset{\;|\;\theta \;|\;-1}{\underset{m=0}{\sum }}\frac{\psi_{0}^{m}}{m!}t_{n+1}^{m}+\frac{1}{\Gamma \left(\theta \right)}\overset{n}{\underset{q=0}{\sum }}b_{q,n+1}f\left(t_{q},\psi_{h}\left(t_{q}\right)\right), \end{array}$$

with

(43) $$\begin{array}{c} b_{q,n+1}=\frac{h^{\theta }}{\theta }\left({\left(n+1-q\right)}^{\theta }-{\left(n-q\right)}^{\theta }\right). \end{array}$$

The error estimate is

(44) $$\begin{array}{c} \underset{0\leq q\leq k}{\max}\left|\psi \left(t_{q}\right)-\psi_{h}\left(t_{q}\right)\right|=O\left(h^{p}\right), \end{array}$$

with *k* ∈ *ℕ* and *p* = min(2, 1 + *θ*).

### 4.1. Application of the ABM Method to the Proposed Model

In this subsection, we solve numerically the nonlinear fractional model using the ABM method. In view of the generalized ABM method, the numerical scheme for the proposed model (18) is given in the following form [36]:

(45) $$\begin{array}{c} s_{h}\left(t_{n+1}\right)=s_{h0}+\frac{h^{\theta }}{\Gamma \left(\theta +2\right)}f_{s_{h}}\left(t_{n+1},s_{h}^{P}\left(t_{n+1}\right),e_{h}^{p}\left(t_{n+1}\right),a_{h}^{p}\left(t_{n+1}\right),i_{h}^{p}\left(t_{n+1}\right),s_{v}^{P}\left(t_{n+1}\right),e_{v}^{p}\left(t_{n+1}\right),i_{v}^{p}\left(t_{n+1}\right)\right)+\frac{h^{\theta }}{\Gamma \left(\theta +2\right)}\overset{n}{\underset{q=0}{\sum }}a_{q,n+1}f_{s_{h}}\left(t_{q},s_{h}\left(t_{q}\right),e_{h}\left(t_{q}\right),a_{h}\left(t_{q}\right),i_{h}\left(t_{q}\right),s_{v}\left(t_{q}\right),e_{v}\left(t_{q}\right),i_{v}\left(t_{q}\right)\right),\\ e_{h}\left(t_{n+1}\right)=e_{h0}+\frac{h^{\theta }}{\Gamma \left(\theta +2\right)}f_{e_{h}}\left(t_{n+1},s_{h}^{P}\left(t_{n+1}\right),e_{h}^{p}\left(t_{n+1}\right),a_{h}^{p}\left(t_{n+1}\right),i_{h}^{p}\left(t_{n+1}\right),s_{v}^{P}\left(t_{n+1}\right),e_{v}^{p}\left(t_{n+1}\right),i_{v}^{p}\left(t_{n+1}\right)\right)+\frac{h^{\theta }}{\Gamma \left(\theta +2\right)}\overset{n}{\underset{q=0}{\sum }}a_{q,n+1}f_{e_{h}}\left(t_{q},s_{h}\left(t_{q}\right),e_{h}\left(t_{q}\right),a_{h}\left(t_{q}\right),i_{h}\left(t_{q}\right),s_{v}\left(t_{q}\right),e_{v}\left(t_{q}\right),i_{v}\left(t_{q}\right)\right),\\ a_{h}\left(t_{n+1}\right)=a_{h0}+\frac{h^{\theta }}{\Gamma \left(\theta +2\right)}f_{a_{h}}\left(t_{n+1},s_{h}^{P}\left(t_{n+1}\right),e_{h}^{p}\left(t_{n+1}\right),a_{h}^{p}\left(t_{n+1}\right),i_{h}^{p}\left(t_{n+1}\right),s_{v}^{P}\left(t_{n+1}\right),e_{v}^{p}\left(t_{n+1}\right),i_{v}^{p}\left(t_{n+1}\right)\right)+\frac{h^{\theta }}{\Gamma \left(\theta +2\right)}\overset{n}{\underset{q=0}{\sum }}a_{q,n+1}f_{a_{h}}\left(t_{q},s_{h}\left(t_{q}\right),e_{h}\left(t_{q}\right),a_{h}\left(t_{q}\right),i_{h}\left(t_{q}\right),s_{v}\left(t_{q}\right),e_{v}\left(t_{q}\right),i_{v}\left(t_{q}\right)\right),\\ i_{h}\left(t_{n+1}\right)=i_{h0}+\frac{h^{\theta }}{\Gamma \left(\theta +2\right)}f_{i_{h}}\left(t_{n+1},s_{h}^{P}\left(t_{n+1}\right),e_{h}^{p}\left(t_{n+1}\right),a_{h}^{p}\left(t_{n+1}\right),i_{h}^{p}\left(t_{n+1}\right),s_{v}^{P}\left(t_{n+1}\right),e_{v}^{p}\left(t_{n+1}\right),i_{v}^{p}\left(t_{n+1}\right)\right)+\frac{h^{\theta }}{\Gamma \left(\theta +2\right)}\overset{n}{\underset{q=0}{\sum }}a_{q,n+1}f_{i_{h}}\left(t_{q},s_{h}\left(t_{q}\right),e_{h}\left(t_{q}\right),a_{h}\left(t_{q}\right),i_{h}\left(t_{q}\right),s_{v}\left(t_{q}\right),e_{v}\left(t_{q}\right),i_{v}\left(t_{q}\right)\right),\\ s_{v}\left(t_{n+1}\right)=s_{v0}+\frac{h^{\theta }}{\Gamma \left(\theta +2\right)}f_{s_{v}}\left(t_{n+1},s_{h}^{P}\left(t_{n+1}\right),e_{h}^{p}\left(t_{n+1}\right),a_{h}^{p}\left(t_{n+1}\right),i_{h}^{p}\left(t_{n+1}\right),s_{v}^{P}\left(t_{n+1}\right),e_{v}^{p}\left(t_{n+1}\right),i_{v}^{p}\left(t_{n+1}\right)\right)+\frac{h^{\theta }}{\Gamma \left(\theta +2\right)}\overset{n}{\underset{q=0}{\sum }}a_{q,n+1}f_{s_{v}}\left(t_{q},s_{h}\left(t_{q}\right),e_{h}\left(t_{q}\right),a_{h}\left(t_{q}\right),i_{h}\left(t_{q}\right),s_{v}\left(t_{q}\right),e_{v}\left(t_{q}\right),i_{v}\left(t_{q}\right)\right),\\ e_{v}\left(t_{n+1}\right)=e_{v0}+\frac{h^{\theta }}{\Gamma \left(\theta +2\right)}f_{e_{v}}\left(t_{n+1},s_{h}^{P}\left(t_{n+1}\right),e_{h}^{p}\left(t_{n+1}\right),a_{h}^{p}\left(t_{n+1}\right),i_{h}^{p}\left(t_{n+1}\right),s_{v}^{P}\left(t_{n+1}\right),e_{v}^{p}\left(t_{n+1}\right),i_{v}^{p}\left(t_{n+1}\right)\right)+\frac{h^{\theta }}{\Gamma \left(\theta +2\right)}\overset{n}{\underset{q=0}{\sum }}a_{q,n+1}f_{e_{v}}\left(t_{q},s_{h}\left(t_{q}\right),e_{h}\left(t_{q}\right),a_{h}\left(t_{q}\right),i_{h}\left(t_{q}\right),s_{v}\left(t_{q}\right),e_{v}\left(t_{q}\right),i_{v}\left(t_{q}\right)\right),\\ i_{v}\left(t_{n+1}\right)=i_{v0}+\frac{h^{\theta }}{\Gamma \left(\theta +2\right)}f_{i_{v}}\left(t_{n+1},s_{h}^{P}\left(t_{n+1}\right),e_{h}^{p}\left(t_{n+1}\right),a_{h}^{p}\left(t_{n+1}\right),i_{h}^{p}\left(t_{n+1}\right),s_{v}^{P}\left(t_{n+1}\right),e_{v}^{p}\left(t_{n+1}\right),i_{v}^{p}\left(t_{n+1}\right)\right)+\frac{h^{\theta }}{\Gamma \left(\theta +2\right)}\overset{n}{\underset{q=0}{\sum }}a_{q,n+1}f_{s_{v}}\left(t_{q},s_{h}\left(t_{q}\right),e_{h}\left(t_{q}\right),a_{h}\left(t_{q}\right),i_{h}\left(t_{q}\right),s_{v}\left(t_{q}\right),e_{v}\left(t_{q}\right),i_{v}\left(t_{q}\right)\right), \end{array}$$

where

(46) $$\begin{array}{c} s_{h}^{p}\left(t_{n+1}\right)=s_{h0}+\frac{1}{\Gamma \left(\theta \right)}\overset{n}{\underset{q=0}{\sum }}b_{q,n+1}f_{s_{h}}\left(t_{q},s_{h}\left(t_{q}\right),e_{h}\left(t_{q}\right),a_{h}\left(t_{q}\right),i_{h}\left(t_{q}\right),s_{v}\left(t_{q}\right),e_{v}\left(t_{q}\right),i_{v}\left(t_{q}\right)\right),\\ e_{h}^{p}\left(t_{n+1}\right)=e_{h0}+\frac{1}{\Gamma \left(\theta \right)}\overset{n}{\underset{q=0}{\sum }}b_{q,n+1}f_{e_{h}}\left(t_{q},s_{h}\left(t_{q}\right),e_{h}\left(t_{q}\right),a_{h}\left(t_{q}\right),i_{h}\left(t_{q}\right),s_{v}\left(t_{q}\right),e_{v}\left(t_{q}\right),i_{v}\left(t_{q}\right)\right),\\ a_{h}^{p}\left(t_{n+1}\right)=a_{h0}+\frac{1}{\Gamma \left(\theta \right)}\overset{n}{\underset{q=0}{\sum }}b_{q,n+1}f_{a_{h}}\left(t_{q},s_{h}\left(t_{q}\right),e_{h}\left(t_{q}\right),a_{h}\left(t_{q}\right),i_{h}\left(t_{q}\right),s_{v}\left(t_{q}\right),e_{v}\left(t_{q}\right),i_{v}\left(t_{q}\right)\right),\\ i_{h}^{p}\left(t_{n+1}\right)=i_{h0}+\frac{1}{\Gamma \left(\theta \right)}\overset{n}{\underset{q=0}{\sum }}b_{q,n+1}f_{i_{h}}\left(t_{q},s_{h}\left(t_{q}\right),e_{h}\left(t_{q}\right),a_{h}\left(t_{q}\right),i_{h}\left(t_{q}\right),s_{v}\left(t_{q}\right),e_{v}\left(t_{q}\right),i_{v}\left(t_{q}\right)\right),\\ s_{v}^{p}\left(t_{n+1}\right)=s_{v0}+\frac{1}{\Gamma \left(\theta \right)}\overset{n}{\underset{q=0}{\sum }}b_{q,n+1}f_{s_{v}}\left(t_{q},s_{h}\left(t_{q}\right),e_{h}\left(t_{q}\right),a_{h}\left(t_{q}\right),i_{h}\left(t_{q}\right),s_{v}\left(t_{q}\right),e_{v}\left(t_{q}\right),i_{v}\left(t_{q}\right)\right),\\ e_{v}^{p}\left(t_{n+1}\right)=e_{v0}+\frac{1}{\Gamma \left(\theta \right)}\overset{n}{\underset{q=0}{\sum }}b_{q,n+1}f_{s_{h}}\left(t_{q},s_{h}\left(t_{q}\right),e_{h}\left(t_{q}\right),a_{h}\left(t_{q}\right),i_{h}\left(t_{q}\right),s_{v}\left(t_{q}\right),e_{v}\left(t_{q}\right),i_{v}\left(t_{q}\right)\right),\\ s_{h}^{p}\left(t_{n+1}\right)=i_{v0}+\frac{1}{\Gamma \left(\theta \right)}\overset{n}{\underset{q=0}{\sum }}b_{q,n+1}f_{i_{v}}\left(t_{q},s_{h}\left(t_{q}\right),e_{h}\left(t_{q}\right),a_{h}\left(t_{q}\right),i_{h}\left(t_{q}\right),s_{v}\left(t_{q}\right),e_{v}\left(t_{q}\right),i_{v}\left(t_{q}\right)\right). \end{array}$$

Further, we have

(47) $$\begin{array}{c} f_{s_{h}}\left(t_{q},s_{h}\left(t_{q}\right),e_{h}\left(t_{q}\right),a_{h}\left(t_{q}\right),i_{h}\left(t_{q}\right),s_{v}\left(t_{q}\right),e_{v}\left(t_{q}\right),i_{v}\left(t_{q}\right)\right)=\mu_{h}-\left(1-\varepsilon_{h}\right)\beta_{v}qci_{v}s_{h}-\mu_{h}s_{h}, \end{array}$$

(48) $$\begin{array}{c} f_{e_{h}}\left(t_{q},s_{h}\left(t_{q}\right),e_{h}\left(t_{q}\right),a_{h}\left(t_{q}\right),i_{h}\left(t_{q}\right),s_{v}\left(t_{q}\right),e_{v}\left(t_{q}\right),i_{v}\left(t_{q}\right)\right)=\left(1-\varepsilon_{h}\right)\beta_{v}qci_{v}s_{h}-m_{1}e_{h}, \end{array}$$

(49) $$\begin{array}{c} f_{a_{h}}\left(t_{q},s_{h}\left(t_{q}\right),e_{h}\left(t_{q}\right),a_{h}\left(t_{q}\right),i_{h}\left(t_{q}\right),s_{v}\left(t_{q}\right),e_{v}\left(t_{q}\right),i_{v}\left(t_{q}\right)\right)=f_{h}\alpha_{h}e_{h}-m_{2}a_{h}, \end{array}$$

(50) $$\begin{array}{c} f_{i_{h}}\left(t_{q},s_{h}\left(t_{q}\right),e_{h}\left(t_{q}\right),a_{h}\left(t_{q}\right),i_{h}\left(t_{q}\right),s_{v}\left(t_{q}\right),e_{v}\left(t_{q}\right),i_{v}\left(t_{q}\right)\right)=\left(1-f_{h}\right)\alpha_{h}e_{h}-m_{3}i_{h}, \end{array}$$

(51) $$\begin{array}{c} f_{s_{v}}\left(t_{q},s_{h}\left(t_{q}\right),e_{h}\left(t_{q}\right),a_{h}\left(t_{q}\right),i_{h}\left(t_{q}\right),s_{v}\left(t_{q}\right),e_{v}\left(t_{q}\right),i_{v}\left(t_{q}\right)\right)=\mu_{v}-\left(1-\varepsilon \right)\beta_{h}ci_{h}s_{v}-\mu_{v}s_{v}-\left(1-\varepsilon_{h}\right)\beta_{h}c\left(1-\eta_{h}\right)a_{h}s_{v}, \end{array}$$

(52) $$\begin{array}{c} f_{e_{v}}\left(t_{q},s_{h}\left(t_{q}\right),e_{h}\left(t_{q}\right),a_{h}\left(t_{q}\right),i_{h}\left(t_{q}\right),s_{v}\left(t_{q}\right),e_{v}\left(t_{q}\right),i_{v}\left(t_{q}\right)\right)=\left(1-\varepsilon \right)\beta_{h}ci_{h}s_{v}-m_{4}e_{v}+\left(1-\varepsilon \right)\beta_{h}c\left(1-\eta_{h}\right)a_{h}s_{v}, \end{array}$$

(53) $$\begin{array}{c} f_{i_{v}}\left(t_{q},s_{h}\left(t_{q}\right),e_{h}\left(t_{q}\right),a_{h}\left(t_{q}\right),i_{h}\left(t_{q}\right),s_{v}\left(t_{q}\right),e_{v}\left(t_{q}\right),i_{v}\left(t_{q}\right)\right)=\alpha_{v}e_{v}-\mu_{v}i_{v}. \end{array}$$

In addition, the quantities

(54) $$\begin{array}{c} f_{s_{h}}\left(t_{n+1},s_{h}^{P}\left(t_{n+1}\right),e_{h}^{p}\left(t_{n+1}\right),a_{h}^{p}\left(t_{n+1}\right),i_{h}^{p}\left(t_{n+1}\right),s_{v}^{P}\left(t_{n+1}\right),e_{v}^{p}\left(t_{n+1}\right),i_{v}^{p}\left(t_{n+1}\right)\right),\\ f_{e_{h}}\left(t_{n+1},s_{h}^{P}\left(t_{n+1}\right),e_{h}^{p}\left(t_{n+1}\right),a_{h}^{p}\left(t_{n+1}\right),i_{h}^{p}\left(t_{n+1}\right),s_{v}^{P}\left(t_{n+1}\right),e_{v}^{p}\left(t_{n+1}\right),i_{v}^{p}\left(t_{n+1}\right)\right),\\ f_{a_{h}}\left(t_{n+1},s_{h}^{P}\left(t_{n+1}\right),e_{h}^{p}\left(t_{n+1}\right),a_{h}^{p}\left(t_{n+1}\right),i_{h}^{p}\left(t_{n+1}\right),s_{v}^{P}\left(t_{n+1}\right),e_{v}^{p}\left(t_{n+1}\right),i_{v}^{p}\left(t_{n+1}\right)\right),\\ f_{i_{h}}\left(t_{n+1},s_{h}^{P}\left(t_{n+1}\right),e_{h}^{p}\left(t_{n+1}\right),a_{h}^{p}\left(t_{n+1}\right),i_{h}^{p}\left(t_{n+1}\right),s_{v}^{P}\left(t_{n+1}\right),e_{v}^{p}\left(t_{n+1}\right),i_{v}^{p}\left(t_{n+1}\right)\right),\\ f_{s_{v}}\left(t_{n+1},s_{h}^{P}\left(t_{n+1}\right),e_{h}^{p}\left(t_{n+1}\right),a_{h}^{p}\left(t_{n+1}\right),i_{h}^{p}\left(t_{n+1}\right),s_{v}^{P}\left(t_{n+1}\right),e_{v}^{p}\left(t_{n+1}\right),i_{v}^{p}\left(t_{n+1}\right)\right),\\ f_{e_{v}}\left(t_{n+1},s_{h}^{P}\left(t_{n+1}\right),e_{h}^{p}\left(t_{n+1}\right),a_{h}^{p}\left(t_{n+1}\right),i_{h}^{p}\left(t_{n+1}\right),s_{v}^{P}\left(t_{n+1}\right),e_{v}^{p}\left(t_{n+1}\right),i_{v}^{p}\left(t_{n+1}\right)\right),\\ f_{i_{v}}\left(t_{n+1},s_{h}^{P}\left(t_{n+1}\right),e_{h}^{p}\left(t_{n+1}\right),a_{h}^{p}\left(t_{n+1}\right),i_{h}^{p}\left(t_{n+1}\right),s_{v}^{P}\left(t_{n+1}\right),e_{v}^{p}\left(t_{n+1}\right),i_{v}^{p}\left(t_{n+1}\right)\right) \end{array}$$

are derived from system (53), at the points *t*_*n*+1_, *n* = 1, 2, 3, ⋯., *m*.

### 4.2. Fractional-Order and Parameter Estimation Using Real Chikungunya Data

In this section, we will utilize the chikungunya data for Colombia (weekly cases observed in 2015) presented in [24] to numerically solve system (18) and determine the best fractional-order parameter *θ* that minimizes the deviations between the real data and model estimates. Data constitute of weekly reported chikungunya cases for Colombia in the year 2015. Despite it being a challenging task, estimation of fractional-order and model parameters is an integral part in mathematical modeling of infectious diseases. Several techniques such as the maximum likelihood iterated filtering and the nonlinear least-squares curve fitting are often used to validate proposed epidemiological models with data.

The fitting process in this paper was done by making use of the least-squares method and Nelder-Mead algorithm [45]. The Nelder-Mead algorithm was used to perform a broad search of the parameter space and is less dependent on initial guesses. Once a good fit was determined, these parameters as the initial guess to search for a more localized region. We fitted the model to cumulative daily new infection data presented in [24]. Since our proposed model constitutes a normalized population, we have normalized the weekly cases by assuming that the total human population in the area where these cases were reported is assumed to be around 19,471,223 [24]. The cumulative new infections predicted by model (18), *C*(*t*), are given by the solution of the following equation:

(55) $$\begin{array}{c} {\;}_{b}^{c}D_{t}^{\theta }C\left(t\right)=\alpha_{h}^{\theta }\left(1-f_{h}\right)e_{h}\left(t\right). \end{array}$$

In order to compute the best fitting, we implemented the function

(56) $$\begin{array}{c} F:{\mathbb{R}}_{\left(\theta ,\eta_{h},\phi ,\varepsilon_{h},\beta_{h}\right)}^{5}⟶{\mathbb{R}}_{\left(\theta ,\eta_{h},\phi ,\varepsilon_{h},\beta_{h}\right)}, \end{array}$$

where *θ*, *η*_*h*_, *ϕ*, *ε*_*h*_, *β*_*h*_ are variables such that

1. for a given (*θ*, *η*_*h*_, *ϕ*, *ε*_*h*_, *β*_*h*_), solve numerically the system of differential equation (18) and equation (55) to obtain a solution ${\hat{Y}}_{i}\left(t\right)=\left({\hat{s}}_{hi},{\hat{e}}_{hi},{\hat{a}}_{hi},{\hat{i}}_{hi},{\hat{s}}_{vi},{\hat{e}}_{vi},{\hat{i}}_{vi}\right)$, which is an approximation of the real-world data *Y*(*t*)
2. Set *t*_0_ = 1 (the fitting process starts in week 1) and for *t* = 2, 3, ⋯, 52, corresponding to weeks in where data are available, evaluate the computed numerical solution for *i*_*h*_(*t*); that is., ${\hat{i}}_{h}\left(2\right)$, ${\hat{i}}_{h}\left(3\right),$…..$,{\hat{i}}_{h}\left(52\right)$
3. Compute the root mean square (RMSE) of the difference between ${\hat{i}}_{h}\left(2\right),{\hat{i}}_{h}\left(3\right),.\cdots ,{\hat{i}}_{h}\left(52\right)$ and observed cases. This function *𝔽* returns the root-mean-square error (RMSE) where

(57) $$\begin{array}{c} \text{ RMSE}=\sqrt{\frac{1}{n}\overset{52}{\underset{k=1}{\sum }}{\left(i_{h}\left(k\right)-{\overset{\wedge }{i}}_{h}\left(k\right)\right)}^{2}} \end{array}$$

(4) Determine a global minimum for the RMSE using Nelder-Mead algorithm

The function *𝔽* takes values in ℝ^5^ and returns a positive real number, the RMSE that measures the closeness of the model predictions to the observed data. On performing the fitting process, we assumed the following initial conditions *e*_*h*_(0) = 0.0002, *a*_*h*_ = *i*_*h*_(0) = 0.0001, *s*_*h*_(0) = 1 − *e*_*h*_(0) − *a*_*h*_(0) − *i*_*h*_(0), *e*_*v*_(0) = 0.0002, *i*_*v*_(0) = 0.0001, and *s*_*v*_(0) = 1 − *e*_*v*_(0) − *i*_*v*_(0) and the baseline values for the model parameters are in Table 1.

Figure 2 depicts the root-mean-square error (RMSE) for different derivative orders. The simulation results show that a global minimum error of estimation for the given data set occurs for *θ* = 0.64 with  RMSE = 2.08 × 10^−7^.  Figure 3 illustrates the model estimates for *θ* = 0.64 and *θ* = 1 (the classical model). From the illustration, one can be able to compare the predictability strength between the integer and fractional models. From the illustrations, we can observe that estimates for the integer model are close to the real data for the first 4 weeks; thereafter, the estimates significantly deviate from the reported cases compared to the estimates of the fractional-order model. Hence, we conclude that the fractional model presents better forecasts compared to the integer model.

Figure 4 shows the simulation of residuals against the predicted values of chikungunya cases in Colombia. It was noted that the residuals did not follow any particular path (exhibited a random pattern), suggesting that the model system (18) was a good fit well to chikungunya cases in Colombia as reported in [24].

### 4.3. Sensitivity of the Reproduction Number to Model Parameters

From the results in Theorems 7 and 8, it is apparent that basic reproduction number *R*_0_ is an integral parameter for chikungunya persistence and extinction in the community; hence, there is a need to determine the sensitivity of *R*_0_ to each parameter. One of the techniques of determining the sensitivity of *R*_0_ to each parameter is through the computation of an elasticity index; that is, for a parameter *ν*, the elasticity index is found by the formula(*ν*/*R*_0_)(*∂R*_0_/*∂ν*). Model parameters that have a positive elasticity index will increase the magnitude of *R*_0_ whenever they are increased while those with negative index will decrease *R*_0_ whenever they are increased. Thus, this linearized sensitivity analysis gives an idea of parameters that are vital in reducing *R*_0_ below unity in order for the disease to die out in the community. Results on computations on the elasticity indices are shown in Figure 5.

From the results in Figure 5, one can observe that the mosquito feeding (biting) rate (parameter *c*) has the largest elasticity index than all the other model parameters that define *R*_0_. In particular, if the mosquitoes increase their feeding rate by 10%, then the magnitude of *R*_0_ will also increase by 10%. Parameters *β*_*h*_ (transmission rate of the disease from humans to mosquito per bite), *β*_*v*_ (transmission rate of the disease from mosquito to human per bite), *ϕ* (the number of mosquitoes per individual), and *μ*_*v*_ (mortality rate of mosquitoes) have a similar elasticity index in absolute value. However, an increase in *β*_*h*_, *β*_*v*_, and *ϕ* will increase the size of *R*_0_ while an increase in *μ*_*v*_ reduces the size of *R*_0_. It is also worth noting that the efficacy of preventative strategies *ε*_*h*_ has a significant effect on reducing the size of *R*_0_. An increase in the efficacy of preventative strategies by 10% will decrease the size of *R*_0_ by 4.28%. From the results, one can conclude that the recovery of symptomatic patients, mortality rate of mosquitoes, and efficacy of preventative strategies are capable of reducing the size of *R*_0_ by a significant margin whenever they are increased.

Simulation results in Figure 6(a) depict the effects of varying mosquito feeding (biting) rate, *c* on *R*_0_. The results show that an increase in mosquito biting rate (modeled by parameter *c*) increases the size of *R*_0_. In particular, whenever *c* > 0.13, then *R*_0_ > 1 which implies that the disease persists in the community.  Figure 6(b) demonstrates the effects of *ε* (efficacy of preventative strategies) on *R*_0_. From the results, we can conclude that whenever the efficacy of preventative strategies is less than 54% all the time, then the disease persists in the community. However, if the reverse is true, it dies off.  Figure 6(c) shows a contour plot of *R*_0_ as a function of *c* and *ε*. We observe that when *c* becomes larger or when *ε* is reduced, *R*_0_ increases, implying a higher disease risk.

Numerical illustrations in Figure 7(a) show the effects of varying mosquito mortality rate, *μ*_*v*_ on *R*_0_. From the results, we note that if the life span of mosquitoes is less than 14 days (*μ*_*v*_ = 0.07 day ^−1^), then the disease dies out, otherwise it persists. In Figure 7(b), we explore the impact of the number of mosquitoes per individuals, *ϕ* on *R*_0_. We can note that whenever the number of vectors per human in the area is greater than 1.3, then the infection persists in the area, otherwise it dies out.

Numerical simulation in Figure 8(a) shows the effects of varying average infectious period for symptomatic patients, 1/*σ*_*h*_ on *R*_0_. From the results, we note that if the average infectious period for symptomatic patients is greater than 40%, the disease dies out, otherwise it persists. In Figure 7(b), we assessed the effect of probability of infection to be transmitted from an infectious mosquito to a susceptible human per bite, *β*_*v*_ on *R*_0_. We can note that whenever the probability of transmission from infectious mosquito to susceptible human is greater than 10%, the disease persists in the area, otherwise it dies out.

### 4.4. Simulation Results to Support Analytical Findings in the Study

In this section, we will carry out numerical simulations so as to support analytical findings in the study. Simulation results in Figure 9 show the convergence of model solutions to the disease-free equilibrium with different derivative orders. We can note that all model solutions converge to the DFE point despite different derivative orders and this is in agreement with Theorem 7. In Figure 10, we can observe that order of the derivative has a significant effect on dynamical behavior on the infected vector and host population over time. In particular, we observe that when the derivative order *θ* is reduced from 1, the memory effect of the system increases, and as a result, the infection grows slowly and the number of infected vectors and host increases over time.

To gain insights on the role of asymptomatic patients on chikungunya dynamics, we simulated model (18) with different values of *f*_*h*_ (proportion of individuals who become asymptomatic patients upon the completion of the incubation period) and the results are shown in Figure 11. The results show that as *f*_*h*_ increases, the exposed human population, asymptomatic patients, and infectious vectors increase remarkably while the infectious human population decreases slightly. Although the exposed vector population increases with increasing *f*_*h*_, the increase is not highly significant compared to the other populations.

To explore the impact of the preventative strategies on long-term dynamics, we simulated model (18) with different values of *ε*_*h*_ with a fixed derivative order (*θ* = 0.64) and the results are in Figure 12. Overall, the results show that as *ε*_*h*_ approaches unity, the disease dies out in the community. In particular, the closer *ε*_*h*_ is to unity, the shorter the time it takes for the disease to become extinct.

## 5. Conclusions

In this paper, we have formulated a mathematical model chikungunya virus transmission that incorporates the human and mosquito populations. The proposed model is based on the Caputo fractional derivative. Fractional calculus has been widely used in mathematical modeling of evolutionary systems with memory effect on dynamics. Previous studies suggest that biological and physical phenomena are characterized by memory effects. Although there are several definitions of fractional derivatives, our choice of using Caputo derivative is as follows: (i) the Caputo derivative for a given function which is constant is zero. Thus, the Caputo operator computes an ordinary differential equation, followed by a fractional integral to obtain the desired order of fractional derivative; (ii) the Caputo fractional derivative allows the use of local initial conditions to be included in the derivation of the model. We computed the model equilibria and determined their existence and global stability. We have shown that the model has two equilibrium points: the disease-free equilibrium (DFE) and the endemic equilibrium (EE), which are both globally stable whenever the reproduction number is less than unity and greater than unity, respectively. We used the 2015 weekly reported cases in Colombia to estimate model parameters. We carried out a comprehensive sensitivity analysis of the model parameters, so as to determine the correlation between the model parameters and the reproduction number. Utilizing results on the sensitivity analysis, we determined threshold values for different model parameters that results in either extinction or persistence of the disease. In particular, this analysis was carried out for model parameters that were found to have a strong correlation with the reproduction number.

The Adams-Bashforth-Moulton method was used to numerically solve the proposed model, and we observed that when the derivative order is reduced from 1, the memory effect of the system increases, and as a result, the infection grows slowly and the number of infected vectors and host increases over time. We believe that our model can provide invaluable insights for public health authorities to predict the effect of chikungunya transmission and analyze its underlying factors and to guide new control efforts.

## Figures and Tables

**Figure 1:** Flow chart for chikungunya disease transmission.

**Figure 2:** The root-mean-square error (RMSE) of the model estimation for different derivative orders. The minimum error estimation is obtained for *θ* = 0.640, and it corresponds to  RMSE = 2.08 × 10^−7^.

**Figure 3:** The estimation of the fractional-order model with *θ* = 0.64 with  RMSE = 2.08 × 10^−7^ and *R*_0_ = 1.53.

**Figure 4:** Simulation of residuals against predicted values of chikungunya cases in Colombia for the model system (18) as reported in [24].

**Figure 5:** Sensitivity analysis of the basic reproduction number *R*_0_ with respect to model parameters. Baseline values used are in Table 1.

**Figure 6:** Effects of varying (a) mosquito feeding (biting) rate, *c* on *R*_0_; (b) the efficacy of preventative strategies, *ε* on *R*_0_; (c) both *ε* and *c* on *R*_0_.

**Figure 7:** Effects of varying (a) mosquito mortality rate, *μ*_*v*_ on *R*_0_, and (b) the number of mosquitoes per individuals, *ϕ* on *R*_0._

**Figure 8:** Effects of varying (a) average infectious period for symptomatic patients, 1/*σ*_*h*_ on *R*_0_, and (b) the probability of infection to be transmitted from an infectious to a susceptible human per bite, *β*_*v*_ on *R*_0_.

**Figure 9:** Dynamical solutions of model (18) with different order derivatives. The solutions were obtained upon setting *ε* = 0.6 giving *R*_0_ = 0.8722. Overall, we can note that as the order of the derivative approaches unity, then time taken by model solutions to converge to the unique DFE equilibrium increases.

**Figure 10:** Dynamical solutions of model (18) with different order derivatives. The solutions were obtained upon setting *ε* = 0.1 giving *R*_0_ = 1.9625. Overall, we observe that when the derivative order *θ* is reduced from 1, the memory effect of the system increases, and as a result, the infection grows slowly and the number of infected vectors and host increases over time.

**Figure 11:** Numerical results for different values of *f*_*h*_ (proportion of individuals who become asymptomatic patients upon the completion of the incubation period) over time with *θ* = 0.64.

**Figure 12:** Numerical results showing the effects of varying *ε*_*h*_ on long-term dynamics of the disease.

**Table 1:** Description of parameters used in the model system (18).

Symbol	Description	Value	Units
*μ*_*h*_	Natural mortality rate of humans	0.00004 day ^−1^	[24]
1/*α*_*h*_	Incubation period of in humans	12 (5–12) days ^−1^	[20, 24]
*c*	Biting rate of human by female mosquito	0.19 (0.19–0.39) days ^−1^	[20, 24]
*f*_*h*_	Proportion of asymptomatic patients	0.1 (0.1–0.3)	[20]
1/*γ*_*h*_	Infectious period for asymptomatic patients	10 (7–10) days ^−1^	[20]
1/*σ*_*h*_	Infectious period for symptomatic patients	7 (7–10) days ^−1^	[20, 24]
*ϕ*	The number of mosquitoes per individuals	3	Fitting
*η*_*h*_	Reduction of infectivity from asymptomatic patients to susceptible mosquito	0.2 (0–1.0)	Fitting
*ε*_*h*_	Efficacy of preventative strategies	0.3 [0–1]	Fitting
*β*_*h*_	Probability of infection to be transmitted from humans to mosquito per bite	0.9 (0.8–1)	Fitting
*β*_*v*_	Probability of infection to be transmitted from an infectious to a susceptible human per bite	0.244 (0.06–0.244)	[24, 46]
1/*μ*_*v*_	Life expectancy of mosquitoes	30 (4–30) day ^−1^	[19, 20]
1/*α*_*v*_	Incubation of mosquitoes	3 (3–7) day ^−1^	[24, 46]
*R*_0_	Basic reproduction number	1.5–7	[20]

## Data Availability

Data used in the model fitting can be obtained free of charge from doi:10.3390/mca24010006. However, the data for parameters used in the model simulation is obtained from the literature, and the references are cited in the manuscript.
